The article "Multiomics Analysis of Genetics and Epigenetics Reveals Pathogenesis and Therapeutic Targets for Atrial Fibrillation" was retracted in 2024. Reasons: signs of a paper mill; suspected computer-generated content; unreliable results or conclusions; concerns about the data.

# Multiomics Analysis of Genetics and Epigenetics Reveals Pathogenesis and Therapeutic Targets for Atrial Fibrillation

**DOI:** 10.1155/2021/6644827

**Published:** 2021-03-25

**Authors:** Li Liu, Jianjun Huang, Baomin Wei, Jianjiao Mo, Qinjiang Wei, Chengcai Chen, Wei Yan, Xiannan Huang, Fengzhen He, Lingling Qin, Hehua Huang, Xue Li, Xingshou Pan

**Affiliations:** ^1^Department of Cardiology, Youjiang Medical University for Nationalities, Affiliated Hospital of Youjiang Medical University for Nationalities, Baise, 533000 Guangxi, China; ^2^Department of Neurology, Youjiang Medical University for Nationalities, Affiliated Hospital of Youjiang Medical University for Nationalities, Baise, 533000 Guangxi, China; ^3^Department of Cardiology, Affiliated Hospital of Youjiang Medical University for Nationalities, Baise, 533000 Guangxi, China; ^4^Department of Ultrasound, Affiliated Hospital of Youjiang Medical University for Nationalities, Baise, 533000 Guangxi, China; ^5^Graduate School of Youjiang Medical University for Nationalities, Baise, 533000 Guangxi, China; ^6^Department of Medical Quality Management, Affiliated Hospital of Youjiang Medical University for Nationalities, Baise, 533000 Guangxi, China; ^7^Department of Anatomy, Youjiang Medical University for Nationalities, Baise, 533000 Guangxi, China; ^8^Department of Electrophysiology, Affiliated Hospital of Youjiang Medical University for Nationalities, Baise, 533000 Guangxi, China

## Abstract

**Objective:**

This study is aimed at understanding the molecular mechanisms and exploring potential therapeutic targets for atrial fibrillation (AF) by multiomics analysis.

**Methods:**

Transcriptomics and methylation data of AF patients were retrieved from the Gene Expression Omnibus (GEO). Differentially expressed genes (DEGs) and differentially methylated sites between AF and normal samples were screened. Then, highly expressed and hypomethylated and lowly expressed and hypermethylated genes were identified for AF. Weighted gene coexpression network analysis (WGCNA) was presented to construct AF-related coexpression networks. 52 AF blood samples were used for whole exome sequence. The mutation was visualized by the maftools package in R. Key genes were validated in AF using independent datasets.

**Results:**

DEGs were identified between AF and controls, which were enriched in neutrophil activation and regulation of actin cytoskeleton. RHOA, CCR2, CASP8, and SYNPO2L exhibited abnormal expression and methylation, which have been confirmed to be related to AF. PCDHA family genes had high methylation and low expression in AF. We constructed two AF-related coexpression modules. Single-nucleotide polymorphism (SNP) was the most common mutation type in AF, especially T > C. MUC4 was the most frequent mutation gene, followed by PHLDA1, AHNAK2, and MAML3. There was no statistical difference in expression of AHNAK2 and MAML3, for AF. PHLDA1 and MUC4 were confirmed to be abnormally expressed in AF.

**Conclusion:**

Our findings identified DEGs related to DNA methylation and mutation for AF, which may offer possible therapeutic targets and a new insight into the pathogenesis of AF from a multiomics perspective.

## 1. Introduction

Atrial fibrillation (AF) is a commonly diagnosed cardiac arrhythmia affecting 1% of the population globally, which is a major risk factor for stroke, heart failure, and premature death [1]. Drugs are the first choice for AF treatment. AF ablation only achieves a success rate of 60-70% [2]. The efficacy of currently available treatments is limited, which increases a major public medical burden and generates a large amount of medical expenses. Moreover, at the molecular levels, the mechanism of AF is incompletely understood. Epidemiological research shows that AF is a complex disease caused by genetic and environmental factors [3]. Due to the limited research on the role of biomarkers in the occurrence and development of AF and the management of clinical AF episodes, it is of importance to explore specific biomarkers of AF.

Multiomics analysis includes genomics (such as whole genome, single-nucleotide polymorphisms (SNP), and copy number alternation (CNA)), expression data (such as mRNA), proteomics, and epigenetics (such as methylation) [4]. With the development of next-generation sequencing (NGS) technology, abnormally expressed genes have been shown to be involved in the pathogenesis of AF [4]. DNA methylation, as one of the main epigenetic modifications, has been confirmed to be related to pathogenesis of AF [5]. DNA methylation occurs at the global and specific gene promoter level. Abnormal DNA methylation can affect the transcription and expression of key regulatory genes [6]. For example, the overall DNA methylation level of the AF group was significantly higher compared to controls [6]. Genome mutations are composed of single-nucleotide variants (SNVs), small insertions-deletions (indels), copy number alterations, and translocations [4]. In recent years, whole exome sequencing studies have identified multiple AF susceptibility gene loci [7]. As an example, a genome-wide association study has identified 104 AF-related genetic variants, which are involved in cardiac structural remodeling [7]. Nevertheless, these genes only partially explain the biological and genetic basis of AF. Only one study identified abnormally expressed genes (PSMC3, TINAG, and NUDT) regulated by methylation for AF based on multiomics analysis [5]. Herein, our study is aimed at comprehensively analyzing the genetics and epigenetics of AF, which could provide a new insight into underlying molecular mechanisms and provide therapeutic targets for AF.

## 2. Materials and Methods

### 2.1. Data Collection and Preprocessing

Microarray expression profile of left atrial (LA) myocardium from patients with AF and sinus rhythm (SR; each *n* = 5) was downloaded from the GSE14975 dataset in the Gene Expression Omnibus (GEO) repository (https://www.ncbi.nlm.nih.gov/gds/) [8]. Furthermore, we obtained the microarray expression profile of 14 AF (7 left AF and 7 right AF) and 12 SR (6 left SR and 6 right SR) samples from the GSE79768 dataset [9]. Methylation profiling data of 11 left atrium samples from 7 AF patients and 4 normal patients were retrieved from the GSE62727 dataset [10]. Microarray expression profile of 3 AF blood samples and 3 normal samples was retrieved from the GSE64904 dataset. normalizeBetweenArrays in the limma package was used to perform quartile normalization on the above microarray expression data [11]. Genes corresponding to each probe were annotated.

### 2.2. Differential Expression or Methylation Analysis

Differentially expressed genes (DEGs) between AF and SR samples were screened with the cutoff of false discovery rate (FDR) < 0.05 or 0.01 and ∣log_2_fold change (FC) | >1. Furthermore, differentially methylated sites were identified under the threshold of FDR < 0.05 and methylation difference > 0.15.

### 2.3. Functional Enrichment Analysis

Functional enrichment analysis of selected genes including Gene Ontology (GO) and Kyoto Encyclopedia of Genes and Genomes (KEGG) was presented using the clusterProfiler package in R [12]. GO included biological process (BP), cellular component (CC), and molecular function (MF). Adjusted *p* value < 0.05 was significantly enriched.

### 2.4. Weighted Gene Coexpression Network Analysis (WGCNA)

Using the WGCNA package [13], coexpression analysis was presented based on the samples in the GSE79768 dataset. The 5000 genes with the largest expression variation were selected, and the samples were clustered based on the expression of these 5000 genes using the hclust package in R. To satisfy a scale-free network, soft threshold value was determined when independence degree > 0.85. Using the dynamic tree cutting, genes with similar expression patterns were merged into one module. The minimum number of genes in the module was 30. 400 genes were randomly selected from 5000 genes. The correlation in expression between these 400 genes was analyzed, and the results were visualized into a heat map. Then, we analyzed Pearson correlation between each module and clinical traits. In each module, correlation between gene significance (GS) and module membership (MM) was calculated.

### 2.5. Protein-Protein Interaction (PPI) Network

Genes in coexpression modules were imported into the STRING online database (version 11.0; https://string-db.org/) [14]. PPI networks were visualized via the Cytoscape software [15] with the cutoff of 0.2 or 0.3. Core networks were constructed via the molecular complex detection (MCODE) [16]. The top ten hub genes were selected using the cytoHubba plugin in Cytoscape according to the maximal clique centrality (MCC) [17].

### 2.6. Whole Exome Sequencing

Blood samples were obtained from 52 AF patients in the Affiliated Hospital of Youjiang Medical University for Nationalities. Whole exome sequencing was achieved by Wuhan Huada Medical Laboratory Co., Ltd. This study followed the guidelines of the Declaration of Helsinki and got the approval of the Ethics Committee of the Affiliated Hospital of Youjiang Medical University for Nationalities (YYFY-LL-2016-03). All participants provided a written informed consent. The demographic characteristics of AF patients are shown in Table 1. The mutation data of whole exome sequencing were filtered as follows: (1) the mutations with 1000G_EAS < 0.1, (2) homozygous mutations (Otherinfo = “hom”), and (3) the mutation type that had the greatest impact on the same gene in the same sample (impact was high, moderate, and low). Then, the selected mutation data were saved in the mutation annotation format (maf) format. The maftools package in R was utilized to count and visualize the maf file [18].

### 2.7. Statistical Analysis

All statistical analysis was presented by R language v4.0.2 (https://www.r-project.org/). *p* value < 0.05 was considered statistically significant.

## 3. Results

### 3.1. DEGs and Their Potential Functions in AF

In the GSE14975 dataset, box plot results showed that the median expression levels of 5 AF and 5 SR samples were basically at the same level (Figure 1(a)). Under the cutoff of FDR < 0.05 and ∣log_2_FC | >1, 4 DEGs were identified between AF and normal samples (Figure 1(b)). Among them, MCEMP1, LOC100288310, and PARP15 were significantly upregulated and F11 was distinctly downregulated in AF compared to SR (Figure 1(b)). These DEGs could conspicuously distinguish AF from SR (Figure 1(c)). In the GSE79768 dataset, there was almost the consistent median expression level between 7 AF and 6 SR left atrium samples (Figure 1(d)). Totally, 1433 DEGs were screened for AF (Figure 1(e)). Among them, 37 DEGs with FDR < 0.01 were displayed, which could significantly distinguish AF from SR (Figure 1(f)). We further explored underlying biological functions of these 1433 DEGs. As shown in Figure 1(g), these DEGs were distinctly enriched in AF-related biological processes such as neutrophil activation, degranulation, and cell adhesion. KEGG enrichment analysis revealed that regulations of actin cytoskeleton, phagosome, and leukocyte transendothelial migration were significantly enriched by these DEGs (Figure 1(h)).

### 3.2. Identification of Differentially Expressed and Methylated Genes for AF

We analyzed methylation expression profile of 7 AF and 4 normal left atrium samples from the GSE62727 dataset.  Figure 2(a) depicts the density plots of *β* value from these 11 samples following normalization. With the threshold of FDR < 0.05 and methylation difference > 0.15, 104 differentially methylated sites were identified between AF and normal samples (Figure 2(b)). In Figure 2(c), differentially methylated sites can distinguish AF from normal samples. As shown in GO enrichment analysis results, genes corresponding to differentially methylated sites might be involved in regulation of hematopoietic stem cell migration. Following correlation analysis between methylation and transcriptome profiles, 28 differentially expressed and methylated genes were screened for AF. Among them, 5 genes have been reported to be involved in AF development. Among them, RHOA (Figure 2(d)), CCR2 (Figure 2(e)), and CASP8 (Figure 2(f)) were hypomethylated and highly expressed in AF than normal samples. Moreover, SYNPO2L (Figures 2(g) and 2(h)) was hypermethylated and lowly expressed in AF compared to controls.

### 3.3. Differentially Expressed and Methylated PCDHA Family Genes in AF

Among 28 differentially expressed and methylated genes, we found that PCDHA family genes were all hypermethylated and lowly expressed in AF compared to controls. PCDHA family genes had two hypermethylated sites between AF and SR samples, including PCDHA1 (Figures 3(a) and 3(b)), PCDHA2 (Figures 3(c) and 3(d)), PCDHA3 (Figures 3(e) and 3(f)), PCDHA4 (Figures 3(g) and 3(h)), PCDHA5 (Figures 3(i) and 3(j)), and PCDHA6 (Figures 3(k) and 3(l)).

### 3.4. Construction of a Coexpression Network for AF

14 AF (7 left AF and 7 right AF) and 12 SR (6 left SR and 6 right SR) samples from the GSE79768 dataset were employed for constructing a coexpression network for AF. After normalization, the expression levels in all samples tended to be the same (Figure 4(a)). According to the 5000 genes with the largest expression variation, the samples were clustered using the hclust package in R. As shown in Figure 4(b), there was no outlier. The biological interaction network must meet the scale free. In this study, when the soft threshold was 5, the independence degree was up to 0.89 (Figure 4(c)). Further analysis confirmed that the constructed coexpression network satisfied scale free when the soft threshold was 5 (Figure 4(d)). Finally, a total of 21 coexpression modules were identified for AF (Figure 4(e)). Each module was represented by a certain color.  Table 2 lists the number of genes contained in each module. 400 genes were randomly selected from 5000 genes. Gene modules were determined based on the similarity of gene expression. The heat map depicted the high correlation between the expression of these 400 genes (Figure 4(f)).

### 3.5. Identification of AF-Related Coexpression Modules and Hub Genes

We further analyzed the correlation between 21 coexpression modules and different clinical traits. In Figure 5(a), magenta module was significantly correlated to AF (*r* = 0.75 and *p* = 1*e* − 05), SR (*r* = −0.75 and *p* = 1*e* − 05), age (*r* = −0.42 and *p* = 0.03), right AF (AFR; *r* = 0.48 and *p* = 0.01), and left SR (AFR; *r* = −0.55 and *p* = 0.004). Turquoise module had a significant correlation with AF (*r* = 0.66 and *p* = 2*e* − 04), SR (*r* = −0.66 and *p* = 2*e* − 04), gender (*r* = −0.42 and *p* = 0.03), left AF (AFL; *r* = 0.46 and *p* = 0.02), and left SR (SRL; *r* = −0.47 and *p* = 0.01). Thus, above two modules were significantly correlated to AF. Scatter plots showed that genes in magenta (Figure 5(b); *r* = 0.76 and *p* = 1.7*e* − 42) and turquoise (Figure 5(c); *r* = 0.61 and *p* = 3.6*e* − 111) modules were significantly related to AF. The cluster analysis results also indicated that magenta and turquoise modules were correlated with AF (Figure 5(d)). Genes in magenta module were significantly correlated with mesenchymal cell proliferation (Figure 5(e)). Furthermore, genes in turquoise module were distinctly enriched in fatty acid metabolic process (Figure 5(f)).

A PPI network composed of 92 nodes was constructed based on genes in magenta module with the cutoff value of 0.2 (Figure 5(g)). According to the PPI network, two core networks were constructed when score = 19 (Figure 5(h)) and 11.862 (Figure 5(i)). Using the cytoHubba plugin of Cytoscape, we identified the top ten hub genes for magenta module according to the maximal clique centrality (MCC; Figure 5(j)), including LSM5 (degree = 55), MRS2 (degree = 80), AIMP1 (degree = 91), ACTR6 (degree = 89), MFN1 (degree = 70), RWDD3 (degree = 73), CAPZA2 (degree = 70), C11orf30 (degree = 82), CCPG1 (degree = 77), and TRAPPC13 (degree = 67). In Figure 5(k), there was a PPI network including 184 nodes on the basis of genes in turquoise module under the cutoff value of 0.3. When score = 14.667 (Figure 5(l)) and 3 (Figure 5(m)), two core networks were built for turquoise module. According to the MCC, the top ten hub genes were identified for turquoise module (Figure 5(n)), including ACTR2 (degree = 22), MIER3 (degree = 32), CSNK1A1 (degree = 78), BCAP29 (degree = 46), PPP1R2 (degree = 55), ADAM10 (degree = 47), RAPGEF6 (degree = 34), DNAAF2 (degree = 40), TRA2A (degree = 51), and SGPP1 (*n* = 117).

### 3.6. Whole Exome Sequencing Reveals Landscape of Mutation in AF

As shown in Figure 6(a) and Table 3, missense mutation and nonsense mutation were the top two variant classifications. Furthermore, SNP was the most common type of mutations, followed by insert and deletion (Figure 6(b)). Among all single-nucleotide variant (SNV) classifications, C > T was the most frequent mutation type, followed by T > C (Figure 6(c)). Furthermore, we counted the mutation frequencies of each sample and the median value of mutation was 66, as shown in Figure 6(d). In Figure 6(e), missense mutation was the most common mutation frequency, followed by nonsense mutation.  Figure 6(f) displays the top ten mutated genes including MUC4 (71%), PHLDA1 (77%), AHNAK2 (52%), MAML3 (44%), OR2T35 (37%), SHROOM2 (25%), SAGE1 (19%), OPN1LW (19%), FLNA (19%), and FUNDC1 (19%) in AF.

PHLDA1 (in frame deletion; 77%), MUC4 (missense mutation; 71%), AHNAK2 (missense mutation; 52%), MAML3 (frame shift deletion; 44%), and OR2T35 (missense mutation; 37%) were the top five genes with mutation frequency among 52 AF samples (Figure 7(a)).  Figure 7(b) displays the top 30 mutually exclusive and cooccurring genes in AF. PHLDA1 and MUC4 exhibited the highest mutation frequencies in AF (Figure 7(c)).

### 3.7. Validation of Key Genes in AF

The microarray expression profiles from the GSE64904 dataset including 3 AF and 3 SR samples were used for validation of key genes in AF. Firstly, the expression profiles of all samples were normalized (Figures 8(a) and 8(b)). PCA results confirmed that there was a distinct difference between AF and SR samples (Figure 8(c)). Heat map visualized the correlation between AF and SR samples based on the gene expression profiles (Figure 8(d)). Under the cutoff of adjusted *p* < 0.05 and FC > 2, 85 genes were upregulated and 73 were downregulated in AF samples compared to SR samples (Figures 8(e) and 8(f)). As shown in Figure 8(g), these genes could significantly distinguish AF from normal samples.  Figure 8(h) separately visualized the top 20 upregulated and downregulated genes between AF and SR samples. However, there was no statistical difference in expression of AHNAK2, MAML3, MUC4, and PHLDA1 between AF and SR samples (Figure 8(i)). In the GSE14975 dataset, PHLDA1 expression was significantly upregulated in AF samples than normal samples (Figure 8(j)). In the GSE79768 dataset, MUC4 expression was distinctly downregulated in AF compared to SR samples (Figure 8(k)).

## 4. Discussion

AF is a common cardiovascular disease. The underlying mechanisms of AF remain largely unclear. Therefore, it is essential for elucidating the underlying mechanism of AF development. This study explored pathogenesis and therapeutic targets for AF through multiomics analysis of genetics and epigenetics.

Abnormal expression is widely involved in the progression of AF. Thus, we identified DEGs between AF and normal samples in different datasets. In the GSE14975 dataset, 4 DEGs were screened for AF compared to normal samples, including 3 upregulated genes (MCEMP1, LOC100288310, and PARP15) and 1 downregulated gene (F11). However, there is no study concerning all of them in AF. In the GSE79768 dataset, 1433 DEGs were screened for AF. Functional enrichment analysis demonstrated that these DEGs were distinctly enriched in AF-related biological processes such as neutrophil activation, degranulation, and cell adhesion. It has been found that myocardial inflammatory infiltration may be a cause of AF, including neutrophil and inflammation markers [19]. Plasma vascular cell adhesion molecule-1 can predict the risk of postoperative AF [20]. In a population-based cohort study, vascular cell adhesion molecule-1 is in association with new-onset AF [21]. Combining previous studies, these DEGs could be involved in AF development via mediating key biological processes. Our KEGG enrichment analysis revealed that these DEGs were associated with regulation of actin cytoskeleton, phagosome, and leukocyte transendothelial migration. As previous studies, it has been found that several genes could regulate the cytoskeleton arrangement of cardiomyocytes in AF [22]. Atrial autophagic flux could be activated in response to AF [23].

Limited evidence suggests that abnormal DNA methylation may be related to the pathogenesis of AF. In this study, we comprehensively analyzed gene expression and DNA methylation profiles. As a result, we identified 28 differentially expressed and methylated genes for AF. As a recent study, Liu et al. identified abnormally expressed PSMC3, TINAG, and NUDT regulated by methylation for AF [5]. Among 28 differentially expressed and methylated genes, 5 have been reported to be related with AF. RHOA, CCR2, and CASP8 were hypomethylated and highly expressed in AF compared to normal samples. Moreover, SYNPO2L was hypermethylated and lowly expressed in AF than controls. High RHOA expression has been confirmed in leukocytes of AF patients compared to controls [24]. A recent study, CCR2 has been identified as a key gene associated with AF progression [25]. CASP8 is associated with recurrence of arrhythmia after catheter ablation of AF [26]. Intriguingly, we found that PCDHA family genes were all hypermethylated and lowly expressed in AF compared to controls, which might become underlying biomarkers for AF.

WGCNA has been widely applied to explore complex biological processes by construction of gene coexpression networks and functional key modules associated with clinical features, which could provide comprehensive insights into specific diseases or conditions [27]. In this study, WGCNA was used to identify potential mechanisms and biomarkers or therapeutic targets for AF using microarray expression profiles. Totally, 21 coexpression modules were constructed for AF. Among them, two coexpression modules (magenta and turquoise) were significantly associated with AF. Recently, Li et al. identify AF-related coexpression modules and hub genes via WGCNA [27]. Functional enrichment analysis revealed that genes in the two modules were involved in various key biological processes. For example, genes in the magenta module could participate in the proliferation of mesenchymal cells. Interstitial fibrosis plays a key role during AF progression. Fibroblast cells are differentiated from proliferative cardiac mesenchymal progenitor cells [28]. Thus, these genes might be associated with pathophysiological processes of AF. Our data suggested that genes in the turquoise were involved in fatty acid metabolic process. As previous studies, serum fatty acid binding proteins have been considered as potential biomarkers for AF [29]. Fatty acid metabolism-related genes are distinctly correlated to autophagy among patients with chronic AF [30]. Hence, it is of importance to further probe into the functions of these genes in the fatty acid metabolic process.

Previous studies on the mechanism of AF focused on specific pathophysiological functions, and relatively few studies have established a comprehensive regulatory network. Based on magenta and turquoise modules, we separately constructed PPI networks for AF, indicating that there were complex interactions between them. Hub genes usually play a core role in the PPI networks. Herein, we identified ten hub genes for magenta- (LSM5, MRS2, AIMP1, ACTR6, MFN1, RWDD3, CAPZA2, C11orf30, CCPG1, and TRAPPC13) and turquoise-related (ACTR2, MIER3, CSNK1A1, BCAP29, PPP1R2, ADAM10, RAPGEF6, DNAAF2, TRA2A, and SGPP1) PPI networks. Among them, high ADAM10 expression has been confirmed to be in relationship with AF [31]. Nevertheless, most of them remain unclear in AF.

SNPs have been widely found on different AF susceptibility loci [32]. Herein, Whole exome sequencing was performed for 52 AF samples. Our data suggested that SNP (especially C > T and T > C) was the most mutation type for AF, which was consistent with previous studies [33]. MUC4, PHLDA1, AHNAK2, and MAML3 were the most frequently four mutated genes for AF. Their abnormal expression was validated in independent datasets. Nevertheless, at present, no studies have reported their mutations in AF.

Collectively, this study expounded pathogenesis and underlying molecular mechanism for AF. Moreover, we provided promising therapeutic targets for AF, which could be worth further exploring in future studies.

## 5. Conclusion

Through multiomics analysis of genetics and epigenetics, we identified abnormal expressed and methylated genes in multiple datasets. Key coexpression modules were constructed, and hub genes were screened for AF. Furthermore, whole exome sequence revealed mutated genes such as PHLDA1 and MUC4 in AF. Taken together, our study provided possible therapeutic targets and a new insight into the pathogenesis of AF.

## Figures and Tables

**Figure 1:** Screening DEGs for AF and functional enrichment analysis. (a) Box plots showing the expression levels of 5 AF and 5 SR samples from the GSE14975 dataset. Red indicates AF samples and blue indicates SR samples. (b, c) Violin plots and hierarchical clustering heat map depicting 4 DEGs between AF and SR samples. Red dot represents an upregulated gene and green dot represents a downregulated gene in AF. (d) The expression levels of 7 AF and 6 SR left atrium samples were shown from the GSE79768 dataset. Red suggests upregulation, while blue suggests downregulation in AF. (e) Screening 1433 DEGs between AF and SR groups. (f) Heat map showing the difference in expression patterns of 37 DEGs with FDR < 0.01 between the AF and SR groups. (g) GO enrichment analysis results composed of biological process (BP), cellular component (CC), and molecular function (MF) based on 1433 DEGs. (h) KEGG pathway annotation results according to 1433 DEGs.

**Figure 2:** Identification of differentially expressed and methylated genes for AF. (a) The density plots showing *β* values from these 11 samples following normalization in the GSE62727 dataset. Red line indicates normal sample and green line indicates AF sample. (b) Violin plots showing 104 differentially methylated sites between the AF and normal groups. Green dots suggest hypomethylated sites and red dots suggest hypermethylated sites in AF. (c) Heat map demonstrating the methylation differences in differentially methylated sites between the two groups. Differentially expressed and methylated genes between the AF and normal groups, including RHOA (d), CCR2 (e), CASP8 (f), and SYNPO2L (g, h).

**Figure 3:** Differentially expressed and methylated PCDHA family genes in AF. (a, b) PCDHA1, (c, d) PCDHA2, (e, f) PCDHA3, (g, h) PCDHA4, (i, j) PCDHA5, and (k, l) PCDHA6.

**Figure 4:** Construction of a coexpression network for AF via WGCNA. (a) Box plots depicting the expression levels in AF and SR samples from the GSE79768 dataset. (b) Sample clustering to detect outliers. (c) Scale independence and mean connectivity corresponding to difference soft threshold values. (d) Frequency of different *k* values and scale-free topology scale *R*^2^ = 0.89 and slope = −1.47. (e) 21 coexpression modules were merged. Each module was marked by a certain color. (f) Heat map depicting the correlation between the expression of randomly selected 400 genes. The darker the color is, the stronger the correlation is.

**Figure 5:** Identification of AF-related coexpression modules and hub genes. (a) Heat map showing the relationships between 21 modules and different clinical traits. Red cell suggests positive correlation between coexpression module and clinical trait. Green suggests negative correlation between coexpression module and clinical trait. The darker the color is, the stronger the correlation is. (b, c) Scatter plots depicting the correlation between molecular membership in magenta or turquoise modules and gene significance for AF. (d) Heat map showing the correlation between AF and 21 coexpression modules. (e, f) GO enrichment analysis results of genes in magenta or turquoise modules. (g) A PPI network based on genes in magenta module. (h, i) Two core networks for genes in magenta module. (j) The top ten hub genes for magenta module according to MCC. (k) A PPI network based on genes in turquoise module. (l, m) Two core networks for genes in turquoise module. (n) The top ten hub genes for turquoise module according to MCC.

**Figure 6:** Landscape of mutation in AF by whole exome sequencing. (a) The mutation frequency in AF. (b) Variant types. (c) SNV classifications. (d) The distribution of variants in each AF sample. (e) The summary of variant classification. (f) The top 10 mutated genes in AF samples.

**Figure 7:** The most common mutated genes in AF. (a) Oncoplot showing the somatic landscape of 52 AF samples. Genes are sorted by mutation frequency. (b) Triangular matrix displaying the top 30 mutually exclusive and cooccurring genes in AF. Green is indicative of tendency to cooccurrence, while pink is indicative of tendency to exclusiveness. (c) The top 100 genes with mutation frequency. The larger the font is, the higher the mutation frequency is.

**Figure 8:** Validation of key genes in AF. (a, b) Box plots showing the expression levels in AF and SR samples before and after normalization. (c) PCA results confirming the difference between AF and SR samples. (d) Heat map visualizing the correlation between different samples based on the gene expression profile. (e, f) Violin plots and scatter plots showing DEGs between the two groups. (g) Hierarchical clustering analysis results demonstrating the expression patterns of DEGs between the two groups. (h) The top 40 DEGs in AF and SR samples. The expression levels of AHNAK2, MAML3, MUC4, and PHLDA1 were detected between AF and SR samples in the GSE64904 (i), GSE14975 (j), and GSE79768 (k).

**Table 1:** Demographic characteristics of AF patients.

Characteristics	Number
Gender	
Female	13
Male	39
Age	66.20 ± 4.86
Hypertension	
Yes	22
No	30
Diabetes	
Yes	6
No	42
Smoking	
Yes	36
No	16

**Table 2:** The number of genes in each coexpression module.

Module	Number of genes
Black	268
Blue	868
Brown	569
Cyan	71
Green	299
Green yellow	111
Grey	84
Grey 60	49
Light cyan	59
Light green	48
Light yellow	42
Magenta	219
Midnight blue	61
Pink	241
Purple	119
Red	277
Royal blue	30
Salmon	76
Tan	96
Turquoise	1081
Yellow	332

**Table 3:** Mutation types in AF and SR samples.

ID	Summary	Mean	Median
Frame shift deletion	41	0.788	1
Frame shift insert	7	0.135	0
In frame deletion	70	1.346	1
In frame insert	19	0.365	0
Missense mutation	1792	34.462	33.5
Nonsense mutation	1391	26.75	28
Nonstop mutation	20	0.385	0
Splice site	58	1.115	1
Translation start site	1	0.019	0
Total	3399	65.365	66

## Data Availability

The datasets analyzed during the current study are available from the corresponding author on reasonable request.

## Abbreviations

AF: Atrial fibrillation
GEO: Gene Expression Omnibus
DEGs: Differentially expressed genes
WGCNA: Weighted gene coexpression network analysis
SNP: Single-nucleotide polymorphism
CNA: Copy number alternation
SNVs: Single-nucleotide variants
indels: Insertions-deletions
LA: Left atrial
SR: Sinus rhythm
FDR: False discovery rate
FC: Fold change
GO: Gene Ontology
KEGG: Kyoto Encyclopedia of Genes and Genomes
BP: Biological process
CC: Cellular component
MF: Molecular function
GS: Gene significance
MM: Module membership
PPI: Protein-protein interaction
MCODE: Molecular complex detection
MCC: Maximal clique centrality
maf: Mutation annotation format.
